The article "Optimization of Data Mining and Analysis System for Chinese Language Teaching Based on Convolutional Neural Network" was retracted in 2023. Reasons: unreliable results or conclusions; concerns about the data; concerns about the peer review; concerns about the citations.

# Optimization of Data Mining and Analysis System for Chinese Language Teaching Based on Convolutional Neural Network

**DOI:** 10.1155/2021/1148954

**Published:** 2021-12-03

**Authors:** Xi Chen

**Affiliations:** ^1^Department of Literature, Northeast Normal University, Changchun 130024, China; ^2^Changchun Education Collage, Changchun 130033, China

## Abstract

Chinese language is also an important way to understand Chinese culture and an important carrier to inherit and carry forward Chinese traditional culture. Chinese language teaching is an important way to inherit and develop Chinese language. Therefore, in the era of big data, data mining and analysis of Chinese language teaching can effectively sum up experience and draw lessons, so as to improve the quality of Chinese language teaching and promote Chinese language culture. Text clustering technology can analyze and process the text information data and divide the text information data with the same characteristics into the same category. Based on big data, combined with convolutional neural network and K-means algorithm, this paper proposes a text clustering method based on convolutional neural network (CNN), constructs a Chinese language teaching data mining analysis system, and optimizes it so that the system can better mine Chinese character data in Chinese language teaching data in depth and comprehensively. The results show that the optimized k-means algorithm needs 683 iterations to achieve the target accuracy. The average K-measure value of the optimized system is 0.770, which is higher than that of the original system. The results also show that K-means algorithm can significantly improve the clustering effect, optimize the data mining analysis system of Chinese language teaching, and deeply mine the Chinese data in Chinese language teaching, so as to improve the quality of Chinese language teaching.

## 1. Introduction

Chinese language is the language with the longest history and the largest number of users in the world, so Chinese language teaching has been valued by people from all walks of life [1]. With the progress of science and the development of Internet technology, more and more industries begin to combine with information technology for information construction. Relevant literature shows that the number of Internet users accounts for 20% of the world's Internet users, and the Internet penetration rate exceeds 54%, so there is a lot of data and information [2]. In the era of big data, data mining and analysis of Chinese language teaching can effectively sum up experience and draw lessons, so as to improve the quality of Chinese language teaching and carry forward Chinese language culture. Clustering algorithm is a convenient data mining technology without training model, which can retrieve and integrate the huge amount of text information [3]. Convolutional neural network (CNN) is one of the most representative deep learning algorithms [4]. Therefore, combining convolutional neural network and K-means clustering algorithm, this paper proposes a K-means algorithm and constructs and optimizes the Chinese language teaching data mining analysis system based on this algorithm, so as to realize the deep mining of Chinese language teaching data and improve the quality of Chinese language teaching.

The article "Optimization of Data Mining and Analysis System for Chinese Language Teaching Based on Convolutional Neural Network" was retracted in 2023. Reasons: unreliable results or conclusions; concerns about the data; concerns about the peer review; concerns about the citations.

Qi used 5 convolutional neural networks such as HRNet to identify the water body of Poyang Lake to realize flood prediction of Poyang Lake [5]. The results show that HRNet can effectively suppress the speckle noise of the image and improve the accuracy of prediction. Fischer et al. proposed a two-thermocouple method based on one-dimensional convolutional neural network to obtain more accurate dynamic temperature and finally realize the dynamic temperature measurement in industrial production. The experimental results show that the fitting degree of the method reaches 96.49%, which is better than the traditional method [6]. Bragazzi et al. proposed a new method of nuclear segmentation by using deep convolutional neural network in order to segment the nucleus accurately in digital pathological images [7]. The research shows that the method can achieve the same or better performance as other latest methods in the public nuclear histopathological dataset. Xia et al. trained a convolutional neural network (CNN) based on the mask area to measure the crown and height of Chinese fir in artificial forest. The results show that the accuracy of the method to the measure crown reaches 84.68% and has a high precision [8]. Based on deep learning, combined with stochastic forest algorithm (RF) and convolutional neural network, Tafti et al. constructed a performance prediction model to predict the performance of membrane electrode assembly (MAE) in PEMFC. The results show that the prediction curve of the model is more fit with the actual curve [9]. Combined with one-dimensional convolutional neural network (OD CNN) and long-term memory (LSTM), a prediction model was designed by Grattarola and Alippi to predict the production of municipal solid waste in Shanghai. The results show that the prediction accuracy of the model is high and has high practicability [10].

Miles et al. used convolutional neural network to identify and diagnose cervical spondylosis and ossification of cervical posterior longitudinal ligament (OPLL) in order to prevent the occurrence of spinal cord injury or traumatic myelopathy in the elderly. The results showed that the accuracy of convolutional neural network reached 86%, which had high practicability [11]. Based on the public data of Iowa, Saeed and Zeebaree used the improved k-prototype clustering algorithm combined with BP neural network to build the prediction model of the recidivism rate after the criminals were released from prison. The research results show that the prediction accuracy of the model is as high as 87.9% [12]. Çolak used hierarchical clustering algorithm and principal component analysis to classify multiple carbon sources and then studied the effect of different fermentation conditions on the fatty acid composition of Trichosporon F1-2 single cell oil [13]. Jouppi et al. used DBSCAN clustering algorithm for data clustering and proposed a new method to improve the web domain recommendation system. The research results show that the probability of the system correctly identifying user pages is 99% [14]. Halverson et al. discussed the relationship between K-means clustering algorithm and principal component analysis (PCA) and proposed two methods combined with K-means and PCA. The results show that the clustering results obtained by the two methods are highly interpretable [15]. An and Qi Yan combined the density-based clustering method and discrete element method (DEM) to build a model to simulate the change of the number and size of fragments produced in the process of ball milling with time. The research results show that the model has high accuracy and practicability [16]. From the above, in recent years, many experts and scholars have made a lot of research achievements in clustering algorithm and convolutional neural network. Clustering algorithm and convolutional neural network are also widely used, but few people apply clustering algorithm and convolutional neural network to Chinese teaching.

The article "Optimization of Data Mining and Analysis System for Chinese Language Teaching Based on Convolutional Neural Network" was retracted in 2023. Reasons: unreliable results or conclusions; concerns about the data; concerns about the peer review; concerns about the citations.

This paper creatively combines convolutional neural network, feedback neural clustering algorithm, and K-means clustering algorithm and proposes a CK-TC algorithm. The algorithm can learn the semantic relationship between Chinese words and sentences on the basis of large-scale corpus, convert the text information into original vectors, and then express words and sentences in the form of word vectors. Convolutional neural network can train and learn the characteristics of these original vectors, construct text vectors, cluster these text vectors by using the optimized k-means algorithm, and finally construct and optimize the Chinese teaching data mining and analysis system.

## 2. Data Mining and Analysis System for Chinese Language Teaching

In the background of big data age, the teaching methods and research directions of Chinese language teaching have changed greatly. The data mining of Chinese language teaching is carried out comprehensively and carefully so that the data mining and analysis system of Chinese language teaching can be established, which can optimize the teaching mode, improve the teaching efficiency, and also make the Chinese language teaching develop scientifically and in the long term.

The meaning of data mining is as follows: the process of extracting valuable information from a large number of fuzzy, noisy, and random data information. The main tasks of data mining can be divided into two categories, namely, data description and prediction [17]. Description refers to finding a way to describe data from a large amount of data and then describing a certain characteristic of data information; prediction is based on the existing data to infer and then make a prediction [18]. The basic steps of data mining are shown in Figure 1.

The main content of Chinese language teaching is Chinese characters, so the data mining of Chinese characters is very important, which can directly reflect the quality and efficiency of Chinese teaching.

## 3. Construction and Optimization of Data Mining Analysis System for Chinese Language Teaching

### 3.1. Chinese Language Data Mining Technology Based on CNN Algorithm

In this paper, CNN is used to extract the feature vectors of Chinese language data, K-means algorithm is used to process and analyze the extracted feature vectors, and then a Chinese language teaching data mining system based on K-means algorithm is constructed.

Generally speaking, the original text data information is not structured data, so it cannot be directly analyzed by data mining algorithm. Therefore, we need to transform the original text data into structured data so that the data mining algorithm can cluster them. The process of transforming original text data into structured data is called text information data preprocessing. Generally speaking, the preprocessing of Chinese text data usually includes word segmentation operation and stop word removal operation [19].

Participle refers to the segmentation of a continuous original text according to some rules, which makes it a set of independent words. Word segmentation is the basis of processing the Chinese text data. Word segmentation is to divide the continuous text information into *n* independent words, words or phrases, and take these independent words, words or phrases, as the basis of feature extraction. Unlike western texts, Chinese text does not have spaces to separate words and sentences, so word segmentation is more difficult. After word segmentation, any element in the set can be extracted as feature items, but independent character vectors are sparse, dimensions are high, and processing is difficult. In Chinese, individual words usually have multiple meanings, so they have great limitations. However, although the phrase has more complete information than individual Chinese characters, it is difficult for the same phrase to appear in many Chinese language texts at the same time, and there are also problems of high and sparse feature vector dimensions, which makes it difficult to calculate the similarity between texts. Therefore, when extracting the features of Chinese text data, words are generally selected as feature items. On the premise of sufficient information, they also have lower feature vector dimension [20].

The article "Optimization of Data Mining and Analysis System for Chinese Language Teaching Based on Convolutional Neural Network" was retracted in 2023. Reasons: unreliable results or conclusions; concerns about the data; concerns about the peer review; concerns about the citations.

Stop words are words that have no practical meaning and make little contribution to text categorization or even have a negative effect. Generally speaking, stop words can be divided into two categories, namely, weak part of speech words and conjunctions or prepositions. Some commonly used stop words are shown in Table 1.

Preprocessing of Chinese language data is one of the most important steps. The effect of preprocessing will directly affect the effect of text clustering and then affect the effect of Chinese language data mining [21].

To make computer understand human language, we need to quantify natural language and map it into a new space. Low dimensional spatial representation can solve the problem of dimension disaster more effectively and mining the potential correlation attributes between words and improves the effectiveness of vector semantics. Therefore, low dimensional spatial representation is used to map natural language to quantitative space. The vector representation of all words is obtained by using the continuous word bag model (CBOW) in word2vcc. CBOW model can predict the current words according to the context of the words [22], as shown in Figure 2.

In Figure 2, *W*_*t*_ stands for the word to be predicted; *W*_*t*_ ± *N* are 2*n* words around the word to be predicted. Using *E* (*W*_*t*_) ± *n*), the demonstrative word *W*_*t*_ ± *N* corresponding to the vector, the word can be predicted. The word vector dimension is set in the input layer, and the vectors corresponding to 2*n* words are connected to form a 2*n* word vector × M-dimensional vector. The hidden layer uses the tanh function as the activation function to initialize the bias term. The output layer uses softmax function to normalize the output value. The neural network structure model of CBOW is shown in Figure 3.

According to CBOW model, all words can be converted into corresponding word vectors, and the vectors contain enough information [23]. For the text features of vectors, convolutional neural network is used to extract the text features. The topology of convolutional neural network is shown in Figure 4.

The article "Optimization of Data Mining and Analysis System for Chinese Language Teaching Based on Convolutional Neural Network" was retracted in 2023. Reasons: unreliable results or conclusions; concerns about the data; concerns about the peer review; concerns about the citations.

Let *x*_*i*_ ∈ *R*^*k*^ be the dimension vector corresponding to the first word in a text, then its value represents the word vector obtained in the previous section, as shown in the following formula:

(1) $$\begin{array}{c} x_{i}=e\left(W_{i}\right). \end{array}$$

Then, a length *n* can be expressed as the following formula:

(2) $$\begin{array}{c} x_{1:n}=x_{1}⊕x_{2}⊕\cdots ⊕x_{n}. \end{array}$$

In formula (2), *x*_*i*:*j*_ represents the join of the words *x*_*i*_, *x*_*i*+1_,…, *x*_*j*_, and *c*_*i*_=*f*(*w* · *x*_*i*:*i*+*h*−1_+*b*) represents the join operator. Convolution kernel *w* ∈ *R*^*hk*^ can generate new features in a window constructed by *h* words, as shown in the following formula:

(3) $$\begin{array}{c} c_{i}=f\left(w\cdot x_{i:i+h-1}+b\right). \end{array}$$

In formula (3), *c*_*i*_ is a new feature obtained by convolution operation on the window formed by the word set *c*=[*c*_1_, *c*_2_, ⋯, *c*_*n*−*h*+1_]; *b* is the offset parameter, which is a real number; *S*(*C*)=∑_*i*=1_^*k*^*S*(*C*_*i*_) is a nonlinear function. The convolution kernel is applied to each word window in the text to obtain a feature plane, as shown in the following formula:

(4) $$\begin{array}{c} c=\left[c_{1},c_{2},\cdots ,c_{n-h+1}\right]. \end{array}$$

K-means algorithm is a clustering algorithm with simple operation and fast convergence speed, which can adjust the clustering results through continuous iteration. K-means algorithm in text clustering, the objective function based on cosine similarity, is shown in the following formula:

(5) $$\begin{array}{c} S\left(C\right)=\sum_{i=1}^{k}S\left(C_{i}\right). \end{array}$$

In formula (5), *C* is a cluster set. *S*(*C*_*i*_) is the similarity of clustering within the cluster and satisfies the following formula:

(6) $$\begin{array}{c} S\left(C_{i}\right)=\left\|F\left(C_{i}\right)\right\|. \end{array}$$

In formula (6), ${\overset{⌢}{c}}_{i}$ is the compound vector of *z*=*z*′∘*r*. Using k-means algorithm, the feature vectors extracted by convolutional neural network can be analyzed and processed, and then clustering operation can be realized. According to the above content, we can build the data mining analysis system of Chinese language teaching.

### 3.2. Optimization of Algorithm Based on CNN and Feedback Neural Network

K-means algorithm can obtain text semantics more effectively, but there are still some defects, so it needs to be optimized. Firstly, convolutional neural network is difficult to find a suitable window size when convolution operation is carried out with a fixed size window: if the window is too large, the training amount of the model will increase and the training effect will decrease. If the window is too small, information will be lost [24–26]. To optimize CNN, the mining effect of Chinese language teaching data mining analysis system is not ideal and needs to be further optimized. Firstly, the convolutional neural network (CNN) is used to learn the pre- and postsemantics of words and expand the word vector. Convolutional neural network is the superposition of forward and backward recurrent neural networks. The output of the whole neural network depends on the state of the hidden layer of the two recurrent neural networks. The general structure of convolutional neural network is shown in Figure 5.

The article "Optimization of Data Mining and Analysis System for Chinese Language Teaching Based on Convolutional Neural Network" was retracted in 2023. Reasons: unreliable results or conclusions; concerns about the data; concerns about the peer review; concerns about the citations.

After the word vector is expanded, the fixed convolution kernel window will not lose the context of the context, so the difficulty of training is reduced. In order to solve the over-fitting problem of traditional convolutional neural network and improve the generalization performance of neural network, dropout algorithm is used to optimize the whole connection layer of the network. The output value of the fully connected layer can be expressed as the following formula:

(7) $$\begin{array}{c} z^{\prime }=\left[{\overset{⌢}{c}}_{1},{\overset{⌢}{c}}_{2},\ldots ,{\overset{⌢}{c}}_{m}\right]. \end{array}$$

In formula (7), ${\overset{⌢}{c}}_{i}$ represents the maximum value of a feature plane and the corresponding feature of convolution kernel. According to Bernoulli distribution theory, the feature vectors input into the clustering algorithm are shown in the following formula:

(8) $$\begin{array}{c} z=z^{\prime }\circ r. \end{array}$$

In formula (8), *C*_*d*_ represents the multiplication operation according to elements, and *d* represents the binary vector obtained according to Bernoulli distribution, as shown in the following formula:

(9) $$\begin{array}{c} r∼\text{Bernoulli}\left(p\right). \end{array}$$

According to formulas (8) and (9), parameters of neural network model can be obtained.

In addition, the clustering effect of K-means algorithm will be affected by the selection of initial clustering center, and it is easy to fall into local optimum in the iterative process [27–29]. In this paper, the feedback neural algorithm is used to optimize it, and the feedback clustering K-means (FCA-K-means) neural algorithm is constructed. After the iteration, the text *d*, the distance from the nearest cluster center is calculated as the following formula:

(10) $$\begin{array}{c} J_{d}^{\left(1\right)}=\left\|d-H\left(C_{d}\right)\right\|. \end{array}$$

In formula (10), *C*_*d*_ includes *d* and *H*(*C*_*d*_) indicates the center of *C*_*d*_. The calculation method of the distance from *d* to the second nearest cluster center is shown in the following formula:

(11) $$\begin{array}{c} J_{d}^{\left(2\right)}=\left\|d-H\left(C_{d}^{\prime }\right)\right\|. \end{array}$$

In formula (10), *C*_*d*_′ is the nearest cluster of *d* and *H*(*C*_*d*_′) expresses the center of *C*_*d*_′. Formula (12) is used to solve the problem where *d* is defined by the concentration.

(12) $$\begin{array}{c} K_{d}=\frac{J_{d}^{\left(2\right)}-J_{d}^{\left(1\right)}}{J_{d}^{\left(1\right)}},\;J_{d}^{\left(1\right)}\neq 0. \end{array}$$

In formula (12), *K*_*d*_ is the concentration of the text to *d*. The definition of clustering result concentration is shown in the following formula:

(13) $$\begin{array}{c} K=\sum_{d\in D}K_{d}. \end{array}$$

In formula (13), *K* represents the concentration of clustering results. According to the above, the loss function of convolutional network can be obtained, as shown in the following formula:

(14) $$\begin{array}{c} L=\sum_{d\in D}\frac{J_{d}^{\left(1\right)}}{J_{d}^{\left(2\right)}-J_{d}^{\left(1\right)}}. \end{array}$$

To avoid the occurrence of *J*_*d*_^(2)^ − *J*_*d*_^(1)^=0, modify formula (14) to the following formula:

(15) $$\begin{array}{c} L=\sum_{d\in D}\frac{J_{d}^{\left(1\right)}}{\max\left(J_{d}^{\left(2\right)}-J_{d}^{\left(1\right)},\varepsilon \right)}. \end{array}$$

In formula (15), *ε* is a minimum greater than 0. After defining the loss function, the clustering effect can be optimized. According to the above content, we can complete the optimization of K-means algorithm, build CK-TC-OP algorithm, and then complete the optimization of Chinese language teaching data mining analysis system.

The article "Optimization of Data Mining and Analysis System for Chinese Language Teaching Based on Convolutional Neural Network" was retracted in 2023. Reasons: unreliable results or conclusions; concerns about the data; concerns about the peer review; concerns about the citations.

## 4. Performance Analysis of Optimized K-Means Algorithm Data Mining Analysis System

### 4.1. Clustering Optimization Effect Analysis of Chinese Text Data

The clustering effect of the traditional K-means algorithm will be affected by the selection of the initial clustering center. The appropriate initial clustering center can improve the clustering effect, while the inappropriate initial clustering center will reduce the clustering effect [30]. Therefore, it is easy to fall into the local optimum in the iterative process, resulting in the reduction of the training effect. In order to solve this problem, the feedback neural algorithm is used to optimize the traditional K-means algorithm and build FCA-K-means. In order to verify the optimization effect of the FCA-K-means, the k-means algorithm model and the FCA-K-means model are constructed, respectively. The same 10000 text data are used to train and test the two models, and the training efficiency of the two models is recorded and compared. The comparison results are shown in Figure 6.

As can be seen in Figure 6, with the increase of the number of iterations, the accuracy of K-means algorithm model and FCA-K-means model is constantly approaching the target accuracy (0.001), and the error is constantly decreasing, but the downward trend of the error curve of FCA-K-means model is obviously faster than that of K-means algorithm model. Among them, K-means algorithm model needs 2193 iterations to approach the target accuracy, while FCA-K-means model only needs 683 iterations, 1510 times less than k-means algorithm model [31]. The above results show that the feedback neural algorithm can effectively optimize the K-means clustering algorithm and improve the clustering effect and training effect.

### 4.2. K-Means Algorithm Optimizes the Mining Effect of Data Mining Analysis System

In natural language processing, K-measure is often used as an evaluation index to evaluate the effect of natural language processing. In order to verify the mining and analysis effect of the optimized Chinese language teaching data mining and analysis system, the optimized Chinese language teaching data mining and analysis system (system 1) and the unoptimized Chinese language teaching data mining and analysis system (system 2) are constructed, respectively. The same parameters are set for the optimized and the unoptimized Chinese language teaching data mining analysis system, that is, the convolution kernel window size of the convolutional neural network is win_ size = 6, 7, 8. The corresponding convolution kernel number num = 150; using the same 10000 sample data, we test the unoptimized Chinese language teaching data mining analysis system and the optimized Chinese language teaching data mining analysis system and record and compare the K-measure values of the two systems under different amounts of sample data, so as to compare the mining effect of the two systems on Chinese language teaching data. The test results of the two systems are shown in Figure 7.

As can be seen from Figure 7, the K-measure values of the two systems increase slowly with the increase of the number of samples. When the number of sample data is 2500, the K-measure value of system 1 is 0.753, and that of system 2 is 0.679, which is 0.074 lower than that of system 1. When the number of sample data is 5000, the K-measure value of system 1 is 0.757, and that of system 2 is 0.683, which is 0.074 lower than that of system 1. When the number of sample data is 7500, the K-measure value of system 1 is 0.776, and that of system 2 is 0.698, which is 0.078 lower than that of system 1. When the number of sample data is 10000, the K-measure value of system 1 is 0.792, and the K-measure value of system 2 is 0.725, which is 0.067 lower than that of system 1. The average K-measure value of system 1 is 0.770, and that of system 2 is 0.696, which is 0.074 lower than that of system 1. The above results show that the optimized Chinese language teaching data mining analysis system has better effect on Chinese language data mining and can achieve Chinese language clustering more deeply and comprehensively, so as to conduct in-depth mining and analysis of Chinese language and improve the quality of Chinese language teaching.

The article "Optimization of Data Mining and Analysis System for Chinese Language Teaching Based on Convolutional Neural Network" was retracted in 2023. Reasons: unreliable results or conclusions; concerns about the data; concerns about the peer review; concerns about the citations.

### 4.3. Analysis of Influencing Factors of Mining Effect

This paper studies and analyzes the factors influencing the mining effect of the data mining analysis system for Chinese language teaching. Firstly, the number of convolution kernels is fixed and the window sizes of convolution kernels are set to win_ size = 3, 4, 5; win_ Size = 6, 7, 8; and win_ Size = 9, 10, 11. Compare the K-measure values of the system under several window sizes, as shown in Figure 8.

As can be seen in Figure 8, generally speaking, the larger the window is, the larger the K-measure value of the data mining and analysis system for Chinese language teaching is. When the number of sample data is 10000, the window size is win_. The K-measure value of size = 9, 10, 11 is 0.792. Set the window size to win_ Size = 3, 4, 5. Compare the K-measure values of the system under different convolution kernel numbers, as shown in Figure 9.

As can be seen from Figure 9, in general, the more convolution cores there are, the larger the K-measure value of the Chinese language teaching data mining and analysis system will be. When the number of sample data is 10000, the K-measure value of the Chinese language teaching data mining and analysis system with num = 150 convolution kernels is 0.763, which is 0.009 larger than that of the Chinese language teaching data mining and analysis system with num = 128 convolution kernels. From the above, we can see that the performance of Chinese language teaching data mining analysis system is positively related to the size of convolution kernel window and the number of convolution kernels. In data mining, we can adjust the size of window and the number of convolution kernels appropriately to ensure the optimal mining effect.

## 5. Discussion

From the above results, it can be seen that the optimized k-means algorithm has higher clustering efficiency, which shows that it has better effect in Chinese language mining and can mine useful data and information more quickly. After the system is optimized by using feedback neural algorithm and cyclic neural network, the F-measure value of the system is significantly improved, which shows that the feedback neural algorithm and cyclic neural network have obvious optimization effect on the system and can effectively improve the performance of the system. When the window size remains unchanged and the number of convolution cores increases, or the number of convolution cores remains unchanged and the window size increases, the F-measure value of the system increases significantly. Therefore, in data mining, the window size and the number of convolution cores can be adjusted appropriately to ensure the optimal mining effect.

The article "Optimization of Data Mining and Analysis System for Chinese Language Teaching Based on Convolutional Neural Network" was retracted in 2023. Reasons: unreliable results or conclusions; concerns about the data; concerns about the peer review; concerns about the citations.

## 6. Conclusion

In this paper, a CK-TC algorithm is proposed by combining convolutional neural network, feedback neural clustering algorithm, and K-means clustering algorithm. The algorithm can learn the semantic relationship between Chinese words and sentences on the basis of large-scale corpus, convert the text information into original vectors, and then express words and sentences in the form of word vectors. Convolutional neural network can train and learn the characteristics of these original vectors, construct text vectors, cluster these text vectors by using the optimized k-means algorithm, and finally construct and optimize the Chinese teaching data mining and analysis system. The results show that the optimized k-means algorithm only needs 683 iterations to achieve the target accuracy, which is 1510 times less than the traditional K-means algorithm model. The average *K*-measurement value of system 1 is 0.770, and the average *K*-measurement value of system 2 is 0.696, which is 0.074 lower than that of system 1. The experimental results show that the performance of Chinese teaching data mining and analysis system is positively correlated with the size of convolution kernel window and the number of convolution kernels.

The above results show that the optimization effect of Chinese teaching data mining and analysis system is good, and it can effectively mine and analyze Chinese teaching data. This study mainly discusses the characteristics of Chinese characters, but there is no in-depth study of the characteristics of homework and learning activities in Chinese teaching, which needs further research.

## Figures and Tables

**Figure 1:** The basic steps of data mining.

**Figure 2:** Basic structure of CBOW model.

**Figure 3:** Neural network structure model of CBOW.

**Figure 4:** Topological structure of convolutional neural networks.

**Figure 5:** The general structure of convolutional neural networks.

The article "Optimization of Data Mining and Analysis System for Chinese Language Teaching Based on Convolutional Neural Network" was retracted in 2023. Reasons: unreliable results or conclusions; concerns about the data; concerns about the peer review; concerns about the citations.

**Figure 6:** Comparison of training efficiency between two models.

**Figure 7:** Test results of two systems.

**Figure 8:** The K-measure value of the system under several window sizes.

**Figure 9:** K-measure values of systems with different convolution kernels.

**Table 1:** Partial stop words.

a	ai	an	an zhao	ba
bei	ben zhe	bici	biru	bing
bie	biren	bian	budan	bici

## Data Availability

The data used to support the findings of this study are available from the author upon request.
